# Stem Cell-Associated Signatures Help to Predict Diagnosis and Prognosis in Ovarian Serous Cystadenocarcinoma

**DOI:** 10.1155/2023/4500561

**Published:** 2023-04-30

**Authors:** Li Li, Weiwei Zhang, Jinxin Qiu, Weiling Zhang, Mengmeng Lu, Jiaqian Wang, Yunfeng Jin, Qinghua Xi

**Affiliations:** ^1^Department of Obstetrics and Gynecology, Affiliated Hospital of Nantong University, Nantong, Jiangsu 226001, China; ^2^Department of Obstetrics and Gynecology, Affiliated Hospital of Nantong University, Medical School of Nantong University, Nantong, Jiangsu 226001, China; ^3^Department of Gynecology, Nantong Geriatric Rehabilitation Hospital, Nantong, Jiangsu 226001, China; ^4^Department of Obstetrics and Gynecology, Binhai County People's Hospital, Yancheng, Jiangsu 224599, China; ^5^Department of Obstetrics and Gynecology, Qidong Maternal and Child Health Hospital, Nantong, Jiangsu 226200, China

## Abstract

Ovarian serous cystadenocarcinoma (OV) is a fatal gynecologic cancer with a five-year survival rate of only 46%. Resistance to platinum-based chemotherapy is a prevalent factor in OV patients, leading to increased mortality. The platinum resistance in OV is driven by transcriptome heterogeneity and tumor heterogeneity. Studies have indicated that ovarian cancer stem cells (OCSCs), which are chemoresistant and help in disease recurrence, are enriched by platinum-based chemotherapy. Stem cells have a significant influence on the OV progression and prognosis of OV patients and are key pathology mediators of OV. However, the molecular mechanisms and targets of OV have not yet been fully understood. In this study, systematic research based on the TCGA-OV dataset was conducted for the identification and construction of key stem cell-related diagnostic and prognostic models for the development of multigene markers of OV. A six-gene diagnostic and prognostic model (C19orf33, CBX2, CSMD1, INSRR, PRLR, and SLC38A4) was developed based on the differentially expressed stem cell-related gene model, which can act as a potent diagnostic biomarker and can characterize the clinicopathological properties of OV. The key genes related to stem cells were identified by screening the genes differentially expressed in OV and control samples. The mRNA-miRNA-TF molecular network for the six-gene model was constructed, and the potential biological significance of this molecular model and its impact on the infiltration of immune cells in the OV tumor microenvironment were elucidated. The differences in immune infiltration and stem cell-related biological processes were determined using gene set variation analysis (GSVA) and single-sample gene set enrichment analysis (ssGSEA) for the selection of molecular treatment options and providing a reference for elucidating the posttranscriptional regulatory mechanisms in OV.

## 1. Introduction

Ovarian serous cystadenocarcinoma (OV) is a fatal gynecologic cancer with a five-year survival rate of only 46% [1, 2]. Most OV patients are resistant to platinum-based chemotherapy, resulting in increased mortality. Platinum resistance in OV is driven by transcriptome and tumor heterogeneity [3]. A previous study has shown that ovarian cancer stem cells (OCSCs), which are chemoresistant and responsible for disease recurrence and relapse, are enriched by platinum-based chemotherapy [4]. Stem cells are critically involved in the prognosis of OV patients and are key pathology mediators of OV [5]. However, the molecular mechanisms and targets of how stem cell-associated genes affect ovarian serous cystadenocarcinoma have not been fully elucidated. In the last few years, several research studies have proven that many proteins, different dysregulated genes, and some other molecular substances in OV may serve as important diagnostic markers and treatment targets. Considering the key role of stem cells in regulating pathological changes in OV, investigating the clinical and biological significance of stem cell-associated genes in OV may also lead to the advancements in OV molecular diagnosis and antitumor therapy.

This study is aimed at identifying and assessing the multigene markers for molecular diagnosis of OV based on the systematic study of differential stem cell-associated genes in OV. Moreover, the prognostic impact of gene models on OV patients and the underlying molecular mechanisms of immune microenvironment infiltration were also analyzed. Further, this study revealed the underlying functional and molecular pathways of immune infiltration and stem cell-associated gene models based on the CIBERSORT algorithm and GSVA. The stem cell-associated gene diagnostic features were established to help in OV diagnosis and investigate the potential biological and prognostic significance of stem cells by applying the LASSO regression analysis. In addition, a TF-miRNA molecular network targeting the 6-gene model was also constructed to investigate the regulatory mechanism of posttranscriptional and molecular mechanisms underlying OV.

## 2. Methods

### 2.1. Identification of Stem Cell-Related Marker Models

In the TCGA-OV dataset, the differentially expressed genes (DEGs) between OV and healthy control tissue samples were identified based on the absolute value of log2FoldChange of more than 0.5 and a false discovery rate (FDR) of less than 0.05 [6]. The stem cell-related biological properties in OVs were examined by using “stem cells” as the keyword and “C7 IMMUNESIGDB” as the filter condition in the molecular signature database (MSigDB, http://www.gseamsigdb.org/gsea/msigdb/ index. jsp), and 26 stem cell-related gene sets were obtained (Table 1). 200 stem cell-related markers were identified in the GSE23321 dataset using comparative screening [7].

### 2.2. Construction of Stem Cell-Based Diagnosis and Prognosis Model of OV

As a result of the differences in the influence of the stem cell-associated molecular mechanisms, the healthy control and OV patient samples may have different stem cell states. Therefore, it is extremely feasible to construct diagnostic models based on necroptosis-associated genes. The stem cell-related biological properties in OVs were examined by using “stem cells” as the keyword and “C7 IMMUNESIGDB” [6, 8] as the filter condition in MSigDB [6, 7], and 26 stem cell-related gene sets were obtained. 200 stem cell-related markers were identified in the GSE23321 dataset using comparative screening [7].

### 2.3. Molecular Diagnostic Efficacy Evaluation

Single-gene receiver operating characteristic (ROC) curves were plotted using the R package pROC to confirm the robustness of the diagnostic model and to calculate the area under the curve (AUC) [9]. Subsequently, the diagnostic performance of the model based on clinical characteristics such as sex, tumor stage, age, grade, metastatic status, DSS (disease-specific survival), OS (overall survival), and PFI (progression-free interval) was evaluated, revealing the association of six stem cell-related marker models in OV with OV prognosis. Time-dependent ROC curves were constructed using the R package rms for the three genes with the most significant weights obtained from the LASSO model, taking into account age and sex information and then visualized using nomograms. The nomogram was validated by measuring the calibration curves using an internal dataset (training set) and an external dataset (validation set) [10].

### 2.4. Gene Enrichment Analysis

Gene Ontology (GO) enrichment analysis was used for the comprehensive functional enrichment study of genes at different levels in order to gain insight into the biological significance of the six stem cell-related marker models in OV [11]. The GO analysis was conducted at three levels, namely, cellular component (CC), biological process (BP), and molecular function (MF), at which the analysis was done. The renowned Kyoto Gene and Genome Encyclopedia Genomes (KEGG) database provides information on biological processes, genomes, diseases, and drugs [12]. All the significant DEGs were annotated with the GO function using the R package clusterProfiler to identify highly enriched biological processes. The enrichment results were visualized using the R package GO plot, and *p* < 0.05 was considered as the significance threshold for enrichment analysis.

### 2.5. Estimation of Immune Cell Infiltration

The gene sets that represented 28 different immune cell types were screened from the existing literature [13]. The single-sample gene set enrichment analysis (ssGSEA) algorithm from the GSVA R package was used to estimate the number of immunological cells infiltrating both OV and normal tissues. At the same time, the influence of the diagnostic marker on the immune microenvironment under immune cell infiltration in OV was investigated by using the CIBERSORT algorithm for deconvolution of the transcriptome expression data based on the principle of linear support vector regression and estimation of the composition and abundance of immune cells from the mixed cell population [14]. The samples with *p* < 0.05 were filtered out to derive an immune cell infiltration matrix [15, 16].

### 2.6. Gene Set Variation Analysis

GSVA [17] is both a nonparameterized and unsupervised method for gene set analysis that uses transcriptome data for predicting the scores of particular pathways or signatures. GSVA is also used for predicting variations in gene set enrichment using expression datasets. GSVA converts the relevant data from a gene-sample matrix to a gene-sample matrix, allowing the pathway enrichment of each sample to be evaluated. GSVA enables the pathway-centric use of standard research techniques, including survival analysis, cluster analysis, and functional enrichment. At the same time, GSVA was performed between groups using the background set based on “msigdb.v7.0.symbols.gmt” and the phenotype characteristic gene set [18].

### 2.7. Quantitative RT-PCR

Total RNA was isolated from normal tissue and tumor tissue from ovarian serous cystadenocarcinoma patients using TRIzol reagent (Beyotime, China). Then, the RNA from each sample (2 *μ*g) was obtained. Subsequently, PCR reactions were performed on Roche LightCycler 480 PCR system (Roche) using SYBR Green Master (Roche). CT values were calculated for all samples using the 2-*ΔΔ*CT method and normalized using the levels of (GAPDH). The primer pairs for the target genes were the following:

*C19orf33*: forward primer TTACCGCCATGGAGTTCGAC and reverse primer CCCTGAAGTTGGAGGCCTTT

*SLC38A4*: forward primer CCCCACTCACACAGAACAGAG and reverse primer CAGCGCTTTCTTGTCCACAC

*PRLR*: forward primer TTTCTGGATTTTACCGACCGT and reverse primer AGGAGAGTTCTTTAGTTTTGCCA

*CBX2*: forward primer GGCTGGTCCTCCAAACATAAC and reverse primer ATCCTTCAGCTCGGGTTTGG

*INSRR*: forward primer GTGTGTGTCCCGTCTTCGAT and reverse primer TCATCCCGAAGTCCCCGAT

*CSMD1*: forward primer ACTAGCAGCCCTTCTTCTGC and reverse primer CACAGTTCTGACCCTTCGCT

### 2.8. Statistical Analysis

Data preparation and analysis were performed using Microsoft Excel and R software 4.0.2. The Mann-Whitney *U* test (i.e., the Wilcoxon rank sum test) was conducted to assess variance between nonnormally distributed variables, and the independent Student's *t* test was used to identify the significance of statistics for normally distributed variables and to compare two consecutive datasets. The chi-square test or Fisher's exact test was used for comparing and assessing the statistical significance between two sets of categorical variables. The Kruskal-Wallis test was used to compare two or more groups, while the Wilcoxon test was used to compare two groups. The pROC package in R was used to plot ROC curves and obtain AUC to determine the accuracy of the risk scores in determining patient prognosis. All the statistical *p* values were two-sided, and *p* < 0.05 was considered statistically significant.

## 3. Results

### 3.1. Analysis of Hub Stem Cell-Related Differential Genes

The DEGs (|logFC| > 0.5 and Padj < 0.05) were initially analyzed in tumor and normal tissues in the TCGA-OV database, which were demonstrated by volcano plots (Figure 1(a)). The stem cell-related biological properties in OVs were investigated by using “stem cells” as the keyword and “C7 IMMUNESIGDB” as the filter condition in MSigDB to obtain 26 stem cell-related gene sets. 200 stem cell-related markers were identified in the GSE23321 dataset by comparative screening. These gene sets were intersected with DEGs (|logFC| > 0.5 and Padj < 0.05) in tumor tissues and healthy tissues in the TCGA-OV dataset (Figure 1(b)).

### 3.2. Construction of Diagnostic and Prognostic Gene Signatures Using LASSO Regression Analysis

Due to the biological significance of stem cells in tumor growth, a diagnosis and prognosis model for predicting OS in OV patients was constructed based on the above 9 stem cell-related hub genes. First, screening was performed using LASSO regression analysis to determine 6 genes with statistical significance based on the optimal lambda value. Thus, a 6-gene diagnostic model consisting of C19orf33, CBX2, CSMD1, INSRR, PRLR, and SLC38A4 was established by screening. This can play an important role in the process of diagnosing OV. The lambda and min values were computed using the logistic LASSO regression algorithm by specifying the loss function for LASSO to achieve a steady state (Figures 2(a) and 2(b)). Subsequently, the impact of these gene-based diagnostic models on the prognosis and OS of OV was visualized using a forest plot (Figures 2(c)–2(e)).

### 3.3. Expression Profiles of Stem Cell-Related 6-Gene Models

The PCA dimensionality reduction was applied to examine the differences in expression of 6 stem cell-related markers in OV (Figures 3(a) and 3(b)), indicating that the genetic models can help to identify OV patients to a certain extent. The differential expression of 6 stem cell-related markers in OV was significantly represented by box plots (Figure 3(c)). Subsequently, a heatmap was used to represent GSVA based on the immunological nonparametric and unsupervised gene sets that can estimate the scores for immune-related pathways or transcriptome signatures. A heatmap indicated that the stem cell-related marker models demonstrated considerable differences in enrichment between the low-risk group and high-risk group of OV patients (Figure 3(d)).

The expressions of six stem cell-related gene models were further analyzed. The correlations between expressions of different molecules were demonstrated by correlation network graphs and correlation heatmaps (Figures 4(a) and 4(b)). The results indicated a strong relationship between the six molecules, with INSRR, PRLR, and SLC38A4 as the most closely related. Subsequently, the histogram representing the differences in gene expression indicated that C19orf33 and CBX2 were highly expressed in OV tissues relative to normal tissues, while lower expression levels of CSMD1, INSRR, PRLR, and SLC38A4 were observed in OV tissues. In addition, the overall expression levels of C19orf33 and CBX2 were significantly higher than those of the remaining molecules (Figures 4(c)–4(h)). And we examined the expression levels of our selected gene markers using RT-PCR (Figures 5(a)–5(f)). Therefore, it was speculated that among the stem cell-related OV diagnostic gene signatures, C19orf33 and CBX2 have higher potential applications.

### 3.4. Functional Enrichment of Stem Cell-Related Marker Models

Subsequently, a functional enrichment analysis of 6 gene signatures significant for OV diagnosis and identification of poor OS prognosis was performed to understand their potential applications in human health (Figures 6(a)–6(h) and Table 1). The enrichment analysis using GO and KEGG was conducted on 6 gene models for OV identification and prognosis prediction with the terms and pathways having *p* < 0.05 considered significantly enriched. The GO enrichment results from three pathways, namely, BP, CC, and MF, indicated that six stem cell-associated GO terms were found to be shared across all 8 subterranean pairs. BP is enriched during the activation of transmembrane receptor protein tyrosine kinase and in the growth hormone receptor signaling pathway via the JAK-STAT cascade. CC is enriched in the PRC1 complex, endosome lumen, euchromatin, and nuclear ubiquitin ligase complex. MF is enriched during oxidoreductase activity and ferroxidase activity as well as when metal ions are oxidized and electrons are accepted by oxygen. Some studies have demonstrated the driving role of JAK-STAT signaling in the ability of cancer stem cells [19, 20]. At the same time, some studies have indicated that the immune microenvironment, such as T cell activation, can be regulated via JAK/STAT molecular pathway, thereby regulating stem cell growth [21, 22].

### 3.5. Verification of Molecular Diagnostic Efficacy

Single-gene ROC curves were developed using the R package pROC to verify the predictive power of the diagnostic model and calculate AUC. The results indicated that all 6 stem cell-related gene signatures in OV could effectively identify OV samples (AUC > 0.7). The ROC curves of gene signatures for OV were analyzed based on the OS data of OV patients (Figures 7(a)–7(f) and 8(a)), indicating AUC = 0.988 for C19orf33, AUC = 0.736 for CBX2, AUC = 0.604 for CSMD1, AUC = 0.547 for INSRR, AUC = 0.944 for PRLR, and AUC = 0.740 for SLC38A4. The relationship of 6 stem cell-related marker models in OV with OV prognosis was determined by analyzing the 1-, 3-, and 5-year ROC curves of the gene signatures (Figures 8(b)–8(f)). Due to the low diagnostic power of INSRR, further analyses were not performed. A comparison indicated that the gene signature demonstrated better performance in discriminating the 1-year survival prognosis of OV patients.

### 3.6. K-M Survival Analysis and Validation of the Stem Cell-Related Signatures

The K-M survival curves of the stem cell-related markers based on the OS time of TCGA-OV patients are shown in Figures 9 and 10. Figures 9(a)–9(f) represent the survival-related investigation of 242 patient samples with OS data analyzed by LASSO regression analysis, and Figures 10(a)–10(f) represent the validation of survival analysis that included all the TCGA-OV patient sample information. Briefly, a comprehensive comparison indicated that the OS results were consistent. These results suggested that the patients with low expression of CBX2 and PRLR had poor survival prognosis and may serve as protective factors for OV patients. The patients with high expression of C19orf33, SLC38A4, INSRR, and CSMD1 had poor survival prognosis, which may be used as high-risk factors for the prognosis of OV.

### 3.7. Cox Regression Analysis of Stem Cell-Associated Signatures and Clinical Subgroup Variables

The univariate and multivariate Cox regression analyses and clinical subgroup variables indicated that primary therapy outcome, age, and tumor status could be used as prognostic risk factors for OV patients when the expressions of stem cell-associated signatures were included (Figures 11(a) and 11(b) and Table 2). The independent analysis of the role of 6 stem cell-associated signatures on the prognosis of OV patients revealed that CBX2 (HR = 0.867, 95% CI (0.760–0.988)) may be a protective indicator for OV, while INSRR (HR = 0.988, 95% CI (1.267–3.748)) and SLC38A4 (HR = 1.399, 95% CI (1.020–1.920)) may be prognostic risk factors for OV patients (Figures 11(c) and 11(d) and Table 3).

### 3.8. Clinical Variables and Prognostic Analysis

Figure 12 shows the differential expression between samples of different clinical subgroups, namely, lymphatic invasion (Figure 12(a)), tumor residual (Figure 12(b)), tumor status (Figure 12(c)), venous invasion (Figure 12(d)), FIGO stage Figure 12(e), age (Figure 12(f)), histologic grade (Figure 12(g)), and primary therapy outcome Figure 12(h). The immune cell infiltration landscape does not reflect significant differences due to small sample size and other factors. However, it can be hypothesized from the box plot of expression differences in clinical subgroup samples that C19orf33, CSMD1, INSRR, PRLR, and SLC38A4 may be potential risk factors for poor prognosis in OV patients, while CBX2 may be a patient-related protective factor for OV prognosis.

Nomograms were developed for predicting the OS among OV patients based on the RMS library. The prediction performance of the nomogram is gauged by the consistency index of the calibrated graph and is assessed by comparing the probability of nomogram prediction to the probability of observed survival. For each patient, the scores for the corresponding variables were calculated and added. The predicted marginal positivity rate can be estimated from the total score of each patient. The nomograms were developed for predicting OV patient prognosis at 1, 3, and 5 years (Figure 13(d)). As shown in Figure 13(e), the calibration plot indicated an excellent degree of agreement between the nomogram predicted and observed results.

### 3.9. Analysis of Immune Cell Infiltration

To investigate the effect of diagnostic marker models on immune cell infiltration in the OV microenvironment, the composition of immune cells in mixed cells was estimated with the CIBERSORT algorithm, which deconvolutes the transcriptome expression matrix according to linear support vector regression and the principle of abundance. The samples with *p* < 0.05 were filtered out to derive an immune cell infiltration matrix [15]. The respective immune cell infiltration levels in the histograms were assessed using the CIBERSORT algorithm and ssGSEA, showing differences in the levels of various immune cell infiltrations between the low and high expression groups of C19orf33, CBX2, CSMD1, INSRR, PRLR, and SLC38A4 (Figure 14). The results showed that all six stem cell-related markers were significantly associated with the distribution of different types of immune infiltrating cells, especially CBX2 and INSRR (Figures 14(b) and 14(d)).

Further, the correlation between stem cell-related markers and the degree of immune cell infiltration was analyzed to understand the role of genes in infiltrating the OV immune microenvironment, thereby leading to a poor prognosis (Figures 15(a)–15(f)). The results revealed a substantial negative relationship between stem cell-related markers and the infiltration levels of immune cells (Figures 16(a)–16(r) and Table 4). We can observe that the elevated expression of stem cell-associated genes correlates with a decrease in the infiltration of various types of immune cells, with T cell subtypes, macrophages, and dendritic cells showing a significant decrease, exhibiting a wide range of suppression from the innate to the adaptive immune system. In other words, immune cell infiltration in the tumor microenvironment is relatively reduced at high gene expression, indicating that insufficient immune cell infiltration results in rapid tumor progression and poor prognosis.

## 4. Discussion

In the past few years, several research studies have demonstrated that many proteins, dysregulated genes, and other molecular substances in OV may serve as crucial diagnostic and therapeutic targets. Since stem cells are closely tied to the pathological changes in OV, evaluating the clinical and biological significance of stem cell-related genes in OV may also lead to advancements in molecular diagnosis and antitumor therapy of OV. The study of stem cell-related genes and tumor development has gradually become a hot topic of research. They can promote tumor development by regulating immunosuppression, promoting vascular regeneration, and directly enhancing tumor proliferation. Meanwhile, tumors with high expression of stem cell-related genes showed more aggressive ability and malignancy.

A comprehensive study based on the TCGA-OV dataset was conducted for the identification and construction of key stem cell-related diagnostic and prognostic models for the development of multigene markers of OV. The key stem cell-related genes were identified by analyzing the genes differentially expressed in normal and OV tissues. The stem cell-related gene diagnostic signatures were established using machine learning, which can help in OV diagnosis and evaluate the potential biological significance of molecular models and their impact on the infiltration of immune cells in the OV tumor microenvironment. The variations in the immune infiltration and stem cell-related biological pathways were determined using ssGSEA and GSVA. They can help in the selection of molecular treatment options and provide a reference for elucidating the posttranscriptional regulatory mechanisms underlying OA. 26 related pathways were obtained by a comprehensive search of [7] datasets containing 200 stem cell-related genes in MSigDB. A total of 9 differential stem cell-related genes were obtained by the intersection of the genes identified by MSigDB with the OV-related DEGs analyzed by TCGA-OV and GTEx databases. Among these 9 differential stem cell-related genes, a gene model affecting the prognosis and survival of OV patients was developed using LASSO regression analysis based on the OS status and survival time of OV patients. Finally, a 6-gene prognostic model consisting of C19orf33, CBX2, CSMD1, INSRR, PRLR, and SLC38A4 was obtained. Based on the differential gene expression analysis, survival analysis, and multivariate and univariate Cox regression analyses in combination with clinical variables, it was verified that the 6-gene prognostic model can be a potential risk factor for poor prognosis of OV patients. The enrichment analysis using GO and KEGG indicated that the stem cell-related markers may influence the prognosis of OV as the JAK-STAT signaling pathway can play a driving role in affecting the ability of cancer stem cells.

C19orf33 and its closely related markers have significant roles in multifocal and multicentric breast cancer (MMBC) and, therefore, can be used as markers for MMBC [6]. Previous studies have revealed a relationship between the immune microenvironment of gastric cancer and CBX-related prognostic gene signatures. Expression levels of mRNA and protein of CBX2/3 were greatly increased in gastric cancer patients. However, the mRNA and protein expression levels of CBX6/7 were lower compared to CBX2/3 [23]. The binding of CBX2 to K27 trimethylated oligonucleosomes has prognostic significance for tumors [24], and CBX2 shapes chromatin accessibility promoting AML via p38 MAPK signaling [25]. CSMD1 is also strongly linked to the occurrence of various tumors and the immune microenvironment [26, 27]. Previous studies have demonstrated that CSMD1 can restrict cancer progression by inhibiting esophageal squamous cell carcinoma proliferation, epithelial-mesenchymal transition, chemotherapy resistance, and inducing immunosuppression [28]. Several studies have shown that INSRR is an insulin receptor-related protein that can enhance the proliferation of several human breast cancer cell lines, possibly because of its synergistic effect with estrogen and insulin-like growth factor (IGF) [29, 30]. The role of PRL and PRL receptors (PRLR) in tumor progression and tumorigenesis is well known [31, 32], and several studies have manifested the regulatory involvement of PRLR in medication responsiveness and the prometastatic effect of PRL on breast cancer and other gynecological cancers [33, 34]. In addition, studies have confirmed that SLC38A4 is a prospective biomarker with therapeutic goal that exerts tumor suppressive effects in hepatocellular carcinoma by modulating the Wnt/*β*-catenin/MYC/HMGCS2 axis [35]. It can be observed that the clinical significance of the stem cell-related six-gene risk model established in this study for cancer was verified by most of the experiments.

For further investigation of the independent prognostic factors dependent on the expression of stem cell-related marker models and affecting the OS of OV patients, the univariate and multivariate Cox regression analyses were conducted by combining the multiple clinical variables, indicating that CBX2 (HR = 0.867, 95% CI (0.760–0.988)) may be a protective factor for OV, while INSRR (HR = 2.179, 95% CI (1.267, 3.748)) and SLC38A4 (HR = 1.399, 95% CI (1.020, 1.920)) can be prognostic risk factors for OV. Subsequently, the differences in the gene expression among clinically distinct subgroups were analyzed. The results from this study were found to be consistent and indicated that C19orf33, CSMD1, INSRR, PRLR, and SLC38A4 may be potential risk factors for poor prognosis in OV patients, while CBX2 may be a potential protective factor for OV. C19orf33 and its closely related markers have important roles in MMBC and can be used as markers for MMBC [36].

The influence of the diagnostic marker model on the immune cell infiltration in the OV microenvironment was investigated by estimating the immune cell composition in mixed cells using the CIBERSORT algorithm based on the principle of linear support vector regression and deconvolution of the transcriptome expression matrix [37, 38]. The samples with *p* < 0.05 were filtered out to derive an immune cell infiltration matrix. All the stem cell-related marker models were associated with the differences in the levels of OV immune infiltration cells. Further correlation analysis demonstrated that the stem cell-related markers were mostly negatively linked to the degree of immune cell infiltration, indicating that insufficient immune cell infiltration can lead to rapid tumor progression and poor prognosis.

Therefore, it is speculated that the six-gene risk model consisting of C19orf33, CBX2, CSMD1, INSRR, PRLR, and SLC38A4 is associated with the activation and migration of OV and is a potential biomarker and therapeutic target in OV.

## Figures and Tables

**Figure 1:** Screening and validation of stem cell-related differential genes. (a) Volcano plot of differential gene expression between OV and healthy tissues, where red represents upregulation and blue represents downregulation. (b) Stem cell-related differentially expressed genes in OV.

**Figure 2:** LASSO analysis and forest plot showing multivariate Cox model results for 10 key stem cell-related genes in OV. (a) Visualization of the lambda value of diagnostic marker identified by LASSO logistic regression algorithm. (b) LASSO coefficient spectrum. (c) Forest plot of multivariate Cox regression model results. (d) Receiver operating characteristic (ROC) curves of stem cell-related genes in severe OV patients at 1, 3, and 5 years. (e) Risk heatmap of stem cell-related genes.

**Figure 3:** Comparison of the molecular models for expression differences in OV patients. (a) Differences in expression of 6 stem cell-related markers in OV tissues. (b) PCA for dimensionality reduction of the discriminative features of 6 stem cell-related markers in OV tissues. (c) Box plot showing the expression of 6 stem cell-related genes, indicating the differential expressions of associated markers in OV were significantly different. (d) Heatmap visualizing the GSVA results of enriched gene sets associated with the stem cell-associated markers between high-risk and low-risk groups for predicting worse prognosis in OV patients.

**Figure 4:** Expression of stem cell-associated genes. (a) Network diagram of gene expression correlation. (b) Correlation heatmap of gene expression. (c–h) Histogram of gene expression differences.

**Figure 5:** RT-PCR detection of stem cell-associated genes. (a–f) RT-PCR results for the six selected stem cell-associated genes were performed and quantified. ^∗^*p* < 0.05, ^∗∗^*p* < 0.01, and ^∗∗∗^*p* < 0.001.

**Figure 6:** GO and KEGG enrichment analyses. (a, b) Histogram of GO/KEGG enrichment analysis. (c, d) Bubble diagram of GO/KEGG enrichment analysis. (e, f) Circle diagram of GO/KEGG enrichment analysis. (g) Chord diagram of GO/KEGG enrichment analyses. (h) Transcription factors (TFs) and miRNA expressions of the six stem cell-related markers in OV, where red represents stem cell-related markers, purple represents their associated TFs, and blue represents their targeted miRNAs.

**Figure 7:** Efficacy of molecular models for poor prognosis in OV patients.

**Figure 8:** Efficacy assessment of stem cell-associated gene signatures for overall survival prognosis in OV patients. (a) ROC curve analysis of a gene signature in OV patients. (b–f) Time-dependent ROC curves of a gene signature for 1-, 3-, and 5-year overall survival.

**Figure 9:** K-M survival curves for stem cell-related markers based on TCGA-OV patient survival data. (a) Unfavorable prognosis of patients at low CBX2 expression, and this association was not statistically significant. (b) Poor survival prognosis was observed in patients with high C19orf33 expression, and this association was not statistically significant. (c) Patients with elevated SLC38A4 expression levels had poor survival prognosis, and this association was statistically significant. (d) Poor survival prognosis of patients with high INSRR expression and, this association was statistically significant. (e) Patients with high CSMD1 expression had poor survival prognosis, and this association was not statistically significant. (f) Worse survival prognosis of patients with low PRLR expression, and this association was not statistically significant.

**Figure 10:** Stem cell-related marker model was validated based on the K-M survival analysis of patients in TCGA-OV. (a) Patients with low CBX2 expression had poor survival prognosis, and the association was statistically significant. (b) Patients with high C19orf33 expression had poor survival prognosis, and the association was not statistically significant. (c) Patients with high SLC38A4 expression had poor survival prognosis, and the association was not statistically significant. (d) Patients with high INSRR expression had poor survival prognosis, and the association was not statistically significant. (e) Patients with high CSMD1 expression had poor survival prognosis, and the association was not statistically significant. (f) Patients with low PRLR expression had poor survival prognosis, and the association was not statistically significant.

**Figure 11:** Multivariate and univariate Cox regression analyses of stem cell-related marker models. (a, b) Forest plots of the univariate and multivariate Cox regression analyses of clinical subgroup variables including primary treatment outcome, age, and tumor status. (c, d) Forest plots of univariate and multivariate Cox regression analyses of clinical subgroup variables based on six-gene stem cell-related marker expression levels.

**Figure 12:** Boxplots showing differences in expression among stem cell-related diagnostic and prognostic genes in each clinical subgroup. (a) Lymphatic invasion. (b) Tumor residual. (c) Tumor status. (d) Venous invasion. (e) FIGO stage. (f) Age. (g) Histologic grade. (h) Primary therapy outcome.

**Figure 13:** Clinical variables and prognostic analysis. (a–c) Boxplots showing differences in the expression of stem cell-related diagnostic and prognostic genes in subgroups with different survival outcomes. (d, e) Nomograms and calibration curves for predicting the overall survival of OV patients.

**Figure 14:** Differences in the infiltration of various immune cells in the OV tumor microenvironment between low and high expression groups of stem cell-related markers.

**Figure 15:** Lollipop plot showing the correlation between stem cell-related markers and the infiltration levels of various immune cells in the OV tumor microenvironment.

**Figure 16:** Scatter plot showing the strongest correlations between stem cell-related markers and the degree of immune cell infiltration. (a–l) Scatter plot showing a significant negative correlation between CBX2 and the degree of immune cell infiltration. (m–q) Scatter plot showing a significant negative correlation between C19orf33 and the degree of immune cell infiltration. (r) SLC38A4 indicated a significant negative correlation with the infiltration of aDC.

**Table 1:** GO and KEGG enrichment analyses of stem cell-associated signatures.

Ontology	ID	Description	*p* adjust	*q* value
BP	GO:0007171	Activation of transmembrane receptor protein tyrosine kinase	0.038	0.016
	GO:0060397	JAK-STAT cascade involved in growth hormone signaling pathway	0.038	0.016

CC	GO:0035102	PRC1 complex	0.031	0.012
	GO:0031904	Endosome lumen	0.031	0.012
	GO:0000791	Euchromatin	0.031	0.012
	GO:0000152	Nuclear ubiquitin ligase complex	0.031	0.012

MF	GO:0004322	Ferroxidase activity	0.030	0.008
	GO:0016724	Oxidoreductase activity, oxidization of metal ions with oxygen as acceptor	0.030	0.008

KEGG	hsa04917	Prolactin signaling pathway	0.084	0.050
	hsa04630	JAK-STAT signaling pathway	0.086	0.052

**Table 2:** Clinical subgroup analysis of the univariate and multivariate Cox regression models.

Characteristics	Total (*N*)	Univariate analysis		Multivariate analysis	
		HR (95% CI)	*p* value	HR (95% CI)	*p* value
FIGO stage	374				
Stage I and stage II	24	Reference			
Stage III	293	2.045 (0.905–4.621)	0.085	1.981 (0.712–5.511)	0.190
Stage IV	57	2.495 (1.057–5.889)	0.037	1.750 (0.599–5.111)	0.306
Primary therapy outcome	307				
PD	27	Reference			
SD	22	0.441 (0.217–0.895)	0.023	0.440 (0.211–0.918)	0.029
PR	42	0.652 (0.384–1.107)	0.113	0.602 (0.347–1.047)	0.072
CR	216	0.152 (0.093–0.247)	<0.001	0.179 (0.107–0.299)	<0.001
Age	377				
≤60	206	Reference			
>60	171	1.355 (1.046–1.754)	0.021	1.402 (1.027–1.913)	0.033
Histologic grade	365				
G2	45	Reference			
G3	320	1.224 (0.827–1.811)	0.313		
Tumor status	336				
Tumor free	72	Reference			
With tumor	264	9.576 (4.476–20.486)	<0.001	9.400 (3.793–23.298)	<0.001
Lymphatic invasion	148				
No	48	Reference			
Yes	100	1.413 (0.833–2.396)	0.200		
PRLR	377				
Low	189	Reference			
High	188	1.019 (0.787–1.320)	0.885		
SLC38A3	377				
Low	187	Reference			
High	190	0.961 (0.742–1.244)	0.761		
INSRR	377				
Low	187	Reference			
High	190	1.251 (0.965–1.622)	0.091	0.989 (0.722–1.356)	0.946
CSMD2	377				
Low	189	Reference			
High	188	1.252 (0.966–1.623)	0.090	0.933 (0.680–1.279)	0.665
CBX2	377				
Low	188	Reference			
High	189	0.739 (0.570–0.958)	0.022	0.938 (0.680–1.293)	0.696
C19orf33	377				
Low	187	Reference			
High	190	1.151 (0.889–1.491)	0.287		

**Table 3:** Univariate and multivariate Cox regression analyses of stem cell-associated signatures.

Characteristics	Total (*N*)	Univariate analysis		Multivariate analysis	
		HR (95% CI)	*p* value	HR (95% CI)	*p* value
C19orf38	377	0.981 (0.784–1.227)	0.866		
CBX2	377	0.884 (0.776–1.007)	0.064	0.867 (0.760–0.988)	0.033
CSMD1	377	1.100 (0.470–2.577)	0.826		
INSRR	377	2.202 (1.293–3.750)	0.004	2.179 (1.267–3.748)	0.005
PRLR	377	0.860 (0.661–1.118)	0.259		
SLC38A4	377	1.408 (1.025–1.934)	0.035	1.399 (1.020–1.920)	0.038

**Table 4:** Correlations of stem cell-associated signatures with immune cell distribution.

Biomarker	Immune cells	Cor	*p* value
CBX2	Cytotoxic cells	-0.467	<0.001
	Th1 cells	-0.406	<0.001
	Neutrophils	-0.400	<0.001
	T cells	-0.395	<0.001
	NK CD56dim cells	-0.348	<0.001
	DC	-0.326	<0.001
	CD8 T cells	-0.311	<0.001
	aDC	-0.310	<0.001
	Macrophages	-0.286	<0.001
	iDC	-0.269	<0.001
	TReg	-0.268	<0.001
	B cells	-0.224	<0.001
	NK cells	0.222	<0.001

C19orf33	TFH	-0.240	<0.001
	Th2 cells	-0.235	<0.001
	Tcm	-0.216	<0.001
	NK cells	-0.210	<0.001
	T helper cells	-0.205	<0.001

SLC38A4	aDC	-0.210	<0.001

INSRR	TFH	0.204	<0.001

## Data Availability

All data generated or analyzed during this study are included in this article.
